The article "Effects of the Dectin-2/TNF-α Pathway on Ventricular Arrhythmia after Acute Myocardial Infarction in Mice" was retracted in 2023. Reasons: signs of a paper mill; compromised peer review; unreliable results or conclusions.

# Effects of the Dectin-2/TNF-*α* Pathway on Ventricular Arrhythmia after Acute Myocardial Infarction in Mice

**DOI:** 10.1155/2022/2521816

**Published:** 2022-08-11

**Authors:** Wei Feng, Zhaojun Wang, Leilei Shi

**Affiliations:** ^1^Department of Cardiology, the First Affiliated Hospital, Harbin Medical University, Harbin, Heilongjiang Province, China; ^2^Department of Cardiology, Langfang Fourth People's Hospital, Langfang, China

## Abstract

**Background:**

Inflammatory responses are involved in ischemic injuries and cardiac repair after acute myocardial infarction (AMI). Dectin-2 is a C-type lectin receptor that induces cytokine production and promotes local inflammatory responses.

**Methods:**

Sixty C57BL/6 mice were randomly assigned to a sham-surgery group, AMI group, or AMI + etanercept group, with 20 mice in each group. Programmed electrical stimulation (PES) was used to anesthetized mice to induce ventricular tachycardia. Real-time polymerase chain reaction (PCR) and western blot analysis were adopted to determine the expression and distribution of dectin-2 in heart tissues. The tumor necrosis factor-*α* (TNF-*α*), interferon-gamma (IFN)-*γ*, interleukin (IL) 4, and IL-5 levels in the serum were determined using ELISAs.

**Results:**

The expression of dectin-2 and TNF-*α* was increased in the myocardium in AMI, and the susceptibility to ventricular arrhythmia (VA) was increased. The induction rate of VA was significantly decreased by etanercept. Compared with those in the sham-surgery group, the AMI group showed significantly higher serum TNF-*α* and IFN-*γ* levels and lower IL-4 and IL-5levels.

**Conclusion:**

Dectin-2 intensifies the activation of the TNF-*α* immune reaction through the Th1 differentiation, which may increase vulnerability to VA in AMI.

## 1. Introduction

Acute myocardial infarction (AMI) is a condition of acute ischemic necrosis of the myocardium. Modern medicine suggests that patients with AMI usually exist with a certain degree of the pathological basis for coronary artery disease. At the onset of AMI, patients exhibit a dramatic reduction or interruption of coronary blood supply, which leads to a severe and persistent acute ischemia of the myocardium and eventually myocardial necrosis [1, 2]. Epidemiological studies have shown that the incidence of AMI in China has been on an increasing trend in the past 30 years, and the main influencing factors include economic and social factors and alterations in human lifestyle and dietary structure. The overall AMI mortality showed an increasing trend from 2002 to 2017, with a rapid upward trend from 2005 onwards and AMI mortality in rural areas exceeding the urban average in 2013 [3]. Sudden cardiac death caused by ventricular arrhythmia (VA) becomes the main cause of death after AMI [1]. Myocardial ischemia is one of the most powerful triggers of leukocyte recruitment and activation. Myocardial necrosis causes sterile inflammation characterized by the activation of immune cells associated with the innate and adaptive immune systems [4, 5]. The immune cells probably play cell-specific functions during the cardiac repair process. However, excessive inflammation may cause additional tissue damage and fibrosis and aggravate subsequent functional impairment, leading to heart failure and arrhythmia [6]. Currently, many traditional Chinese medicine (TCM) extracts exhibit beneficial therapeutic effects against AMI, but there are scarce studies on the pathways through which they work to exert their effects. Thus, it is particularly important to explore effective targets, signaling pathways, and their course of action.

The expression of dectin-2 is a C-type lectin receptor. It has been observed in myeloid cells and induces cytokine production by regulating the T-helper 1 (Th1)/Th2 balance to promote the local inflammatory response [7]. Dectin-2 can increase plaque rupture after MI and wound healing and strengthen cardiac remodeling by increasing the interferon-*γ* (IFN-*γ*) level [8]. However, the accurate role of the dectin-2 signaling pathway in VA after AMI has been marginally explored.

Tumor necrosis factor-*α* (TNF-*α*) is a Th1 cytokine that induces the inflammatory cascade and promotes unlimited lipid uptake, foam cell formation, and atherosclerosis progression [9]. Moreover, the significant changes in the electrical properties of these cells indicate that the overexpression of TNF-*α* in the heart leads to the remodeling of ion channels, such as Ca^2+^ channels and K^+^ channels [10], which are the basis for the generation of action potentials and contribute to VA [11]. In this research, the role of the dectin-2/TNF-*α* pathway in VA after AMI was investigated.

## 2. Methods

### 2.1. Animal Studies

C57BL/6 mice (18–22 g, male, 10 weeks old; Shanghai, China) were chosen as samples in this study. Sixty C57BL/6 mice were randomly assigned to a sham-surgery group, AMI group, or AMI + etanercept group, with 20 mice in each group. All experimental protocols were approved by the local animal care and use committee (Animal Experimental Ethics Association of the First Affiliated Hospital of Harbin Medical University). The methods were carried out in line with the revised Animals (Scientific Procedures) Act, as amended in 1986. Etanercept (Pfizer, 12.5 mg/kg) was subcutaneously injected daily for 7 days [12].

### 2.2. Animal Model of AMI

The experimental animals were subjected to permanent ligation of the left anterior descending artery (AMI and AMI + etanercept groups) or a sham operation without ligation [13]. The AMI + etanercept group received 12.5 mg/kg of etanercept (Pfizer) through subcutaneous injection daily for 7 days. Then, 7 days after the AMI, AMI + etanercept, or sham operation, a protocol of programmed electrical stimulation (PES) was performed on the C57BL/6 mice. Then, all mice were sacrificed, and tissue samples were collected.

### 2.3. Programmed Electrical Stimulation (PES)

A protocol of right ventricular stimulation was applied to C57BL/6 [14]. The animals in each group were anesthetized and fixed, and the chest was opened. A bipolar needle electrode was inserted into the peri-infarcted parts of the left ventricle in the mice of the AMI group and AMI + etanercept group, and the electrode was stimulated to induce arrhythmia by PES. A bipolar needle electrode was inserted into the corresponding parts of the mice in the sham group, and the electrode was stimulated to induce arrhythmia by PES. The circumference of S1S2 was 90 ms, 80 ms, and 70 ms for the electrical stimulation. The voltage was 5 V, the ratio was 10 : 1, and the wave width was 2 ms. Atrial and ventricular intracardiac ECG were recorded using a 1.1 F octapolar electrode catheter inserted into the right ventricle via the right jugular vein [15]. The type of interactional arrhythmia that occurred was recorded. Ventricular tachyarrhythmia (VT) was defined as more than three consecutive ventricular beats >600 bpm [16].

### 2.4. Real-Time Polymerase Chain Reaction (PCR)

Quantitative real-time PCR was used to determine the dectin-2 gene expression in heart tissue. The prepared cDNA was increased and quantified using NCSYB GREEN qPCR Master Mix (Harbin Nachuan Biotechnology Co., Ltd., China) with the following primers: forward 5′-GAGTGAGCAGAATTGCGTTG-3′ and reverse 5′-ATTGCCAGTTGCCATTCC-3′. PCR was operated using a real-time thermal cycler system (ABI7500 Fast RealTime PCR System, Applied Biosystems, USA). The PCR amplification procedure started with a single denaturation step at 95°C, lasted for 15 min, and had 40 amplification cycles including denaturation at 95°C for 10 s, followed by annealing at 64°C for 30 s for dectin-2 or annealing at 47.44°C for 30 s for GAPDH. The relative quantification was performed using the 2−ΔΔCt method with GAPDH as a reference [17].

### 2.5. Western Blot Analysis

Dectin-2 protein expression in heart tissue was determined by western blot analysis. Equal amounts of protein samples were loaded, separated by 10% SDS-PAGE, and then transferred to nitrocellulose membranes. The membranes were blocked with TBS-Tween-20 (TBS-T) containing 5% skim milk and incubated overnight at 4°C with an anti-dectin-2 antibody (Abcam, UK). Then, the membranes were incubated with the appropriate anti-dectin-2 secondary antibody (Abcam, Britain). The antibody reactions were detected by an electrochemiluminescence (ECL) kit [18]. The protein levels were analyzed by using NIH Image. The protein levels were normalized to those of GAPDH. Each membrane was incubated with the corresponding internal controls and targeting antibodies. A gel imaging system was used to obtain pictures and analyze the density of the protein bands. The ratio of the density of the target band to that of the internal reference band represented the relative expression level of the target protein. All experiments were repeated at least three times.

### 2.6. ELISA

Blood (2 mL) was collected and centrifuged for 10 min. The expression levels of tumor necrosis factor-*α* (TNF-*α*), interferon-gamma (IFN-*γ*), interleukin (IL) 4, and IL-5 in plasma were determined by ELISA as per the ELISA kit instructions (MILLIPLEX multifactor detection kit, Merck Biotechnology Co., Ltd., Germany). A microplate reader was used to measure the OD value at 450 nm (1510, Thermo, USA), and the concentration was calculated by a standard curve [19].

### 2.7. Immunohistochemistry

To assess the distribution of TNF-*α* and dectin-2, mouse cardiac tissues were paraffinized and sectioned for immunohistochemistry. The tissue sections were dewaxed in C_8_H_10_ and rehydrated in graded ethanol; then, the antigens were retrieved by microwave heating and equilibration in phosphate-buffered saline (PBS), and the slices were treated with 3% hydrogen peroxide to slake endogenous peroxidase activity. Each section was incubated with anti-TNF-*α* and anti-dectin-2 antibodies (Solarbio Bioscience and Technology Co., Ltd., Shanghai, China) after blocking nonspecific areas of the sections, followed by the moderate biotinylated secondary antibody. The slices were stained with diaminobenzidine (DAB) substrate kit (Zhongshan Biology Co., Ltd., China) and then counterstained with hematoxylin briefly. The slices were observed under an Olympus BX53 microscope (Tokyo, Japan) [20].

### 2.8. Statistical Analysis

SPSS 21.0 software for Windows was used for data analyses. The data shown in graphs are expressed as the mean ± standard error (SE). ANOVA and LSD tests were used for pairwise comparisons. A *χ*^2^ test was used to compare the incidence of ventricular arrhythmia after PES between the groups. Differences with a *P* value <0.05 were considered statistically significant.

## 3. Results

### 3.1. Morphological Changes in Myocardial Tissues after AMI

After the hematoxylin and eosin (HE) staining, the myocardial tissues were examined and photographed by microscopy (20x). The results revealed that, in the sham-surgery mice, the myocardial fibers were arranged in an orderly manner without fractures or an enlarged necrotic gap, and the nuclei were fusiform or elliptical. In the AMI and AMI + etanercept mice, myocardial necrosis and the dissolution and fracturing of myocardial fibers with obviously enlarged gaps were observed (Figure 1).

### 3.2. Increased Dectin-2 Expression in AMI

The expression of dectin-2 in the heart tissue was determined via real-time PCR and western blot analysis (Figure 2). Real-time PCR showed that the relative dectin-2 mRNA expression level in the AMI mice and AMI + etanercept mice was higher than that in the sham-surgery mice (*P* < 0.001; Figure 2(a)). The western blot analysis showed higher expression of dectin-2 protein in the AMI mice and AMI + etanercept mice versus that in the sham-surgery mice (*P* < 0.001; Figure 2(b)). The above results suggest highly expressed dectin-2 in AMI.

### 3.3. Increased Expression of TNF-A after AMI

The immunohistochemistry analysis indicated that the expression of dectin-2 in the AMI mice and AMI + etanercept mice was higher than that in the sham-surgery mice (Figure 3(a)). Furthermore, the immunohistochemistry results demonstrated elevated expression of TNF-*α* in the heart tissue of the AMI mice compared with that in the sham-surgery mice (Figure 3(b)). The expression of TNF-*α* in the heart tissue of the AMI + etanercept mice was decreased compared to that in the AMI mice (Figure 3(b)). The above results showed elevated expressions of dectin-2 and TNF-*α* in the heart tissue of the AMI mice. The expression of TNF-*α* was significantly decreased by etanercept.

### 3.4. Increased Vulnerability to VA in the Hearts of AMI Mice Promoted by TNF-*α*

PES was performed in vivo in sham-surgery mice (*n* = 20), AMI mice (*n* = 20), and AMI + etanercept mice (*n* = 20) and induced VT of various beats (Figure 4). No induction of VA occurred in sham-surgery mice (Figure 4(a)). The induction of polymorphic VT occurred in the AMI mice (Figure 4(b)). VA was induced in only 2 of the 20 (10.0%) sham-surgery mice after PES. In contrast, VA was induced in 16 of the 20 (80.0%) AMI mice after PES. VA was induced in 6 of the 20 (30.0%) AMI + etanercept mice after PES. The incidence of VA after PES in the AMI mice was higher than those in the sham-surgery group (*P* < 0.05; Figure 4(c)). Nevertheless, the incidence of VA after PES in the AMI + etanercept mice was lower than in the mice in the AMI (*P* < 0.05; Figure 4(c)). It is suggested that TNF-*α* caused increased vulnerability to VA in the hearts of the AMI mice.

### 3.5. Dectin-2 Boosts TNF-*α* and IFN-*γ* Expression in AMI by Modulating Th1 Differentiation

Dectin-2 plays an important role in inflammation by regulating the Th1/Th2 balance. The inflammatory factor changes in the serum of the AMI, AMI + etanercept, and sham-surgery mice were examined by ELISA (Figure 5). Compared with the sham-surgery mice, the expression level of the TNF-*α* in the AMI mice was significantly increased. Compared with the AMI mice, the expression level of TNF-*α* in the AMI + etanercept mice was significantly decreased (*P* < 0.001; Figure 5(a)). Compared with the sham-surgery mice, the expression level of IFN-*γ* in the AMI and AMI + etanercept mice was significantly increased (*P* < 0.001; Figure 5(b)). Nevertheless, compared with the sham-surgery mice, the level of IL-4 in the AMI and AMI + etanercept mice was significantly decreased (*P* < 0.001; Figure 5(c)). Compared with the sham-surgery mice, the level of IL-5 in the AMI and AMI + etanercept mice was significantly decreased (*P* < 0.001; Figure 5(d)). These results indicate that dectin-2 increases TNF-*α* and IFN-*γ* expression in AMI by modulating Th1 differentiation.

## 4. Discussion

The results showed that the Dectin-2/TNF-*α* pathway promotes VA after AMI. This study involving the sham-surgery, AMI, and AMI + etanercept groups of C57BL/6 mice using PES revealed that the dectin-2/TNF-*α* pathway increases VA after AMI as evidenced by (1) the increased myocardial dectin-2 levels in the AMI mice and (2) increased expression levels of TNF-*α* in the myocardium and increased susceptibility to VA. (3) When TNF-*α* was blocked, the incidence of VA after PES was reduced. (4) Dectin-2 increases TNF-*α* and IFN-*γ* expression by modulating Th1 differentiation after AMI. Therefore, the manipulation of the dectin-2/TNF-*α* pathway may assist in the treatment of VA after AMI. The reason for this result may be that the microcirculation is impaired by vascular endothelial damage and cytokine release after acute myocardial infarction. The dectin-2/TNF-*α* pathway may mediate the release of vasoendothelial reactive substances and reduce vasospasm and thrombotic excess to improve microvascular stability, thereby yielding a positive therapeutic effect in acute myocardial infarction [21].

### 4.1. Increased Dectin-2 Levels in the Myocardium in AMI

Hypoxia and insufficient nutritional supply lead to a marked loss of cardiac tissue, which leads to an inflammatory reaction that initiates cardiac repair processes [22]. However, severe tissue injury is associated with a strong inflammatory response, excessive fibrosis, immune autoreactivity, and hurtful remodeling toward HF [23].

Dectin-2 is a C-type lectin receptor that has a carbohydrate recognition domain for the Ca^2+^-dependent recognition of mannose oligosaccharides. Dectin-2 induces the tyrosine phosphorylation of FcRgamma, activation of NF-*κ*B, internalization of alternative ligands, and upregulation of TNF-*α*, IL-1, IL-12, and IL-23 receptor antagonists to induce an innate immune response [24]. Dectin-2 is found in various myeloid cells and promotes the local inflammatory response. Some studies have examined the presence of dectin-2 signaling in the healing process and cardiac remodeling in cardiovascular diseases and elucidated the underlying molecular mechanisms. Research demonstrated that dectin-2 could increase plague rupture after MI and wound healing and strengthen cardiac remodeling by increasing the IFN-*γ* levels [6]. Dectin-2 is involved in the occurrence of coronary heart disease, has a profound influence on the immune response in the heart, and participates in the pathogenesis of Kawasaki disease. In a Kawasaki disease model, dectin-2 has been shown to mediate the induction of CCL2 production by macrophages in the aortic root and coronary artery-induced vascular inflammation [25]. Therefore, dectin-2 is widely involved in cardiovascular disease and myocardial injury and remodeling through the immune response.

The present study showed that the dectin-2 expression in myocardial tissue in a mouse AMI and AMI + etanercept model was abnormally increased compared with mice in the sham-surgery group, suggesting that the dectin-2 signaling pathway influences the immune response in AMI.

### 4.2. Elevated Expression Levels of TNF-*α* and Susceptibility to VA in AMI

Compared with sham-surgery mice, the expression of TNF-*α* in the myocardium and serum was elevated and that susceptibility to VA was increased in AMI mice. However, the expression of TNF-*α* in the myocardium and serum was decreased, and the incidence of VA after PES was lower in AMI + etanercept mice than that in AMI mice, indicating that TNF-*α* may increase susceptibility to VA in AMI; however, the mechanism by which TNF-*α* causes VA remains unclear.

TNF-*α* inhibits the Ca^2+^ treatment-induced action potential of cardiomyocytes, resulting in a negative inotropic effect and decreased myocardial contractility [26]. These results demonstrated that the action potential duration (APD) of TNF mouse cardiomyocytes was prolonged, the intracellular Ca^2+^ transient species were changed, the Ca^2+^ peak of contraction was decreased, and the Ca^2+^ diastolic peak was increased [27]. These alterations in Ca^2+^ handling cause increased activity and arrhythmia. The dynamic changes in the intercellular coupling, such as the decrease in gap-junction conduction in the presence of high intracellular [Ca^2+^], may also explicate the beginning of re-entrant VT in these mice [28]. Alternatively, alternation in intracellular Ca^2+^-dependent processes via cAMP- or calmodulin-dependent kinases may influence the occurrence of arrhythmia [29].

In addition to abnormal Ca^2+^ treatment, the main reason for APD prolongation is a decreased expression of several K^+^ channels, leading to arrhythmia in TNF mice, which was similar to previous research results. The results showed that the attenuation of transient outward K^+^ current in TNF mice was similar to that reported by Ito in heart failure patients and similar to that in a rat heart failure model and spontaneous arrhythmia [30]. The decrease in the K^+^ current observed in TNF mouse ventricular myocytes seems to contribute partially to the increase in APD that was previously measured with optical localization. Transgenic mice overexpressing the mutant Kv2.x a-subunit had prolonged APD and spontaneous arrhythmia due to a lack of IK and slow2 [11].

The changes in the electrical properties of these marker cells indicate that the overexpression of TNF cells leads to the remodeling of Ca^2+^ plasma channels and the generation of K^+^ channel action potentials, which may lead to VA.

### 4.3. Dectin-2 Increases TNF-*α* and IFN-*γ* Expression by Modulating Th1 Differentiation after AMI

As a C-type lectin receptor, dectin-2 is expressed in various myeloid cells and promotes the local inflammatory response. Dectin-2 triggers the production of many kinds of cytokines and chemokines, with proinflammatory Th1, Th17, and Th2 cytokines included [31]. CD4+ T cells secrete Th1 and Th17 cytokines (such as IFN-*γ*, TNF-*α*, granulocyte-macrophage colony-stimulating factor, and IL-17A), which activate neutrophils, monocytes, macrophages, and dendritic cells to remove fungi [32]. Dectin-2 plays a key role in the protection of Th1 and Th17 cell growth [33]. Dectin-2 induced Th1/Th17 cells to respond to *Candida albicans* and *Aspergillus fumigatus* [34]. Dectin-2-dependent IL-12 production contributes to Th1 differentiation and IFN-*γ* production after *Streptococcus pneumoniae* infection [35]. Dectin-2 is a pattern recognition receptor for fungi, which is selectively expressed on dendritic cells and macrophages [36]. It also recognizes house dust mites (HDMs) and induces cysteinyl leukotriene production by dendritic cells to elicit a Th2 reaction in mouse models, aggravating allergic airway inflammation in mice [37]. Dectin-2 also participates in inflammation responses by regulating the balance of Th1 and Th2 cells. The results demonstrated that the expression of dectin-2 was increased in the mouse AMI model. The expression of TNF-*α* and IFN-*γ* was increased, whereas the levels of IL-4 and IL-5 were decreased in the AMI group. The expression of TNF-*α*, IFN-*γ*, and transcription factors is responsible for Th1 differentiation, and the expression of IL-4, IL-5, and transcription factors is responsible for Th2 differentiation. Interleukin 1*β* (IL-1*β*) promotes the inflammatory response and exacerbates the disease. TNF-*α* is critical in the inflammatory response and is an important mediator of inflammation [38]. This study proposed that dectin-2 increases the potential for TNF-*α* and IFN-*γ* expression to promote the local inflammatory response by modulating Th1 differentiation in a mouse AMI model. IL-1, IL-1*β*, and TNF-1 levels are locally increased, and thus the inhibition of the production of such inflammatory vesicles might be effective in preventing and attenuating the myocardial inflammatory response and protecting myocardial tissue in mice with acute myocardial infarction [39].

Despite ongoing studies on acute myocardial infarction [40, 41], the present study focused on ventricular arrhythmias after AMI and explored the role of the less studied dectin-2/TNF-*α* pathway in mediating inflammatory markers to affect disease prognosis.

## 5. Conclusions

The expression of dectin-2 is increased in the myocardial tissue of AMI mice. Compared with the sham-surgery mice, the expression of TNF-*α* in the myocardium and serum is increased and susceptibility to VA is increased in AMI mice. However, the expression of TNF-*α* in the myocardium and serum is decreased, and the incidence of VA after PES is lower in AMI + etanercept mice than that in AMI mice. The AMI mice showed increased serum levels of TNF-*α* and IFN-*γ* and decreased levels of IL-4 and IL-5. It is possible that dectin-2 increases activation of the TNF-*α*-mediated immune reaction by modulating Th1 differentiation, which may increase vulnerability to VA in the hearts of AMI mice.

## Figures and Tables

**Figure 1:** Morphological changes in sham-surgery, AMI, and AMI + etanercept mice.

**Figure 2:** Dectin-2 levels are increased in the heart after AMI. (a) Dectin-2 mRNA expression in heart tissue was examined by RT-PCR. (b) Dectin-2 protein expression in heart tissue was determined by western blot analysis. Group means were compared using an ANOVA and LSD test for pairwise comparisons. The data are expressed as the mean ± SE. Sham: *n* = 20; AMI: *n* = 20; AMI + etanercept: *n* = 20. ^*∗∗∗*^*P* < 0.001.

**Figure 3:** Expression levels of dectin-2 and TNF-*α* were increased in heart tissue after AMI (a) Expression levels of dectin-2 in heart tissue were examined by immunohistochemistry. (b) Expression levels of TNF-*α* in heart tissue were examined by immunohistochemistry. Sham: *n* = 20; AMI: *n* = 20; AMI + etanercept: *n* = 20.

**Figure 4:** Susceptibility to VA is increased in AMI mice. PES was performed in sham-surgery, AMI, and AMI + etanercept mice. (a) Right ventricular stimulation (atrial and ventricular intracardiac ECG) shows no inducible arrhythmia in a sham-surgery mice with S1, S2, S3, and S4 stimuli. (b) Polymorphic VT in AMI mice induced by S1, S2, S3, and S4 stimuli. (c) PES in 20 sham-surgery, 20 AMI, and 20 AMI + etanercept mice showed susceptibility to VA. *χ*^2^ test was used in 5°C. Sham: *n* = 20; AMI: *n* = 20; AMI + etanercept: *n* = 20. ^*∗*^*P* < 0.05.

**Figure 5:** Effects of dectin-2 on TNF-*α*, IFN-*γ*, IL-4, and IL-5 expression after AMI. ELISA was used to detect inflammatory factors in the serum. (a) TNF-*α*, (b) IFN-*γ*, (c) IL-4, and (d) IL-5 levels in the serum (sham: *n* = 20; AMI: *n* = 20; AMI + etanercept: *n* = 20). Statistical analysis was performed using SPSS 21.0 software. Group means were compared using an ANOVA and LSD test for pairwise comparisons. The data are shown as the mean ± SE. ^*∗∗∗*^*P* < 0.001.

## Data Availability

The datasets used during the present study are available from the corresponding author upon reasonable request.
